# Time series based road traffic accidents forecasting via SARIMA and Facebook Prophet model with potential changepoints

This article has been retracted.

**DOI:** 10.1016/j.heliyon.2023.e22544

**Published:** 2023-11-20

**Authors:** Edmund F. Agyemang, Joseph A. Mensah, Eric Ocran, Enock Opoku, Ezekiel N.N. Nortey

**Affiliations:** a Department of Statistics and Actuarial Science, College of Basic and Applied Sciences, University of Ghana, Ghana; b School of Mathematical and Statistical Science, College of Sciences, University of Texas Rio Grande Valley, USA; c Department of Computer Science, Ashesi University, No. 1 University Avenue, Berekuso, Accra, Eastern Region, Ghana

**Keywords:** Road traffic accident, SARIMA, Facebook Prophet, Potential changepoints, Ghana

## Abstract

Road traffic accident (RTA) is a critical global public health concern, particularly in developing countries. Analyzing past fatalities and predicting future trends is vital for the development of road safety policies and regulations. The main objective of this study is to assess the effectiveness of univariate Seasonal Autoregressive Integrated Moving Average (SARIMA) and Facebook (FB) Prophet models, with potential change points, in handling time-series road accident data involving seasonal patterns in contrast to other statistical methods employed by key governmental agencies such as Ghana's Motor Transport and Traffic Unit (MTTU). The aforementioned models underwent training with monthly RTA data spanning from 2013 to 2018. Their predictive accuracies were then evaluated using the test set, comprising monthly RTA data from 2019. The study employed the Box-Jenkins method on the training set, yielding the development of various tentative time series models to effectively capture the patterns in the monthly RTA data. $SARIMA\;\left(0,1,1\right)\times {\left(1,0,0\right)}_{12}$ was found to be the suitable model for forecasting RTAs with a log-likelihood value of −266.28, AIC value of 538.56, AICc value of 538.92, BIC value of 545.35. The findings disclosed that the $SARIMA\;\left(0,1,1\right)\times {\left(1,0,0\right)}_{12}$ model developed outperforms FB-Prophet with a forecast accuracy of 93.1025% as clearly depicted by the model's MAPE of 6.8975% and a Theil U1 statistic of 0.0376 compared to the FB-Prophet model's respective forecasted accuracy and Theil U1 statistic of 84.3569% and 0.1071. A Ljung-Box test on the residuals of the estimated $SARIMA\;\left(0,1,1\right)\times {\left(1,0,0\right)}_{12}$ model revealed that they are independent and free from auto/serial correlation. A Box-Pierce test for larger lags also revealed that the proposed model is adequate for forecasting. Due to the high forecast accuracy of the proposed SARIMA model, the study recommends the use of the proposed SARIMA model in the analysis of road traffic accidents in Ghana.

## 1 Introduction

The invention of automobiles brought great relief to humanity; people had little complaints due to fatigue from walking long distances, lateness to work and goods and services could be procurred within the shortest possible time [1], [2], [3]. The use of automobiles have increased access to remote places and enhanced livelihood due to related research, promoted social and economic interactions geographically and created jobs [4], [5], [6]. This not withstanding the continuous use and misuse of automobiles have negatively impacted lives as well as property [7]. The rampant occurrence of road accidents seem to have no cure especially in developing countries unlike many studies pertaining to the control and elimination of diseases as reported in the scientific literature [8]. Therefore, many reseachers have given considerable amount of time and space to studying models that could predict the occurrence of road accidents over the years. A study by [9] measured the effects of randomness, exposure, weather, and daylight to variations of road accidents by using a generalized Poisson regression model based on data from four countries (Denmark, Norway, Finland, and Sweden). Their study concluded that randomness and exposure account for eighty to ninety per cent of the variation in road traffic accidents. On the contrary, road accidents are viewed as deterministic occurrences according to a study by [10]. However, inadequate information makes it uncertain how accidents happen. As a result, in this work, we uphold the notion that road accidents are more random than deterministic, as argued by [9], though the vehicle's driver may have a hand in road traffic accidents.

A road traffic accident is a significant cause of death, injury and a disadvantage or handicap worldwide, both in high-income, low-middle income and low-income countries [11]. [12] asserted that “Road Traffic Accidents (RTAs) manifest when a motor vehicle collides with another vehicle, pedestrian, animal, geographical features, or architectural barriers, potentially leading to injuries, property damage, and fatalities”. A host of researchers have commented on the causes of road traffic accidents. [13], among a ton of researchers, attributed the causes to overspeeding, drunk driving, wrong overtaking, poor road network and poor worthiness of many vehicles in the country. Notable causes of RTAs include but not limited to unnecessary speeding, reckless driving, fatigue [14], inadequate experience, traffic rules violation, road surface defects, wrong overtaking, machine failure and defective light [15], [16], overloading, poor vision [17], [18] among others. It is a robust superstitious belief in Africa and Ghana that witches also cause road accidents, as many converted witches and wizards confess and attest to this fact [19], [20]. However, studies have shown that road traffic accidents result from drivers' unethical behaviours [21]. The force behind this could be strongly linked to the inability of the drunk driver to control the vehicle because of sleeping [22]. In addition to drunk drivers, passengers and other drunk road users may not know what happens before, during, and after a road accident. When passengers and other road users behave in such a way, they are prevented from taking action to avoid serious injuries or death. Drivers do what they want and cause accidents that cost lives. The effects of RTAs, apart from causing injuries and death, have also brought about other consequences. Road traffic accidents have been known to cause traumas [23], reduce family or persons involved in the accident's financial position [24], disabilities to people [25], [26] and psychological effects [27] among others. The impact of road accidents has gone far to the extent that some people refuse to drive a vehicle again. RTAs are classified as fatal, serious, or minor based on the damage they inflict on human lives and property [28], [29].

Ghana, classified as a low-middle income earning country, suffers the most regarding road traffic accidents. RTAs are rising each year on Ghana's roads and have become a significant concern for all and sundry in recent times. Even though the road system network in Ghana is terrible, some drivers have also considerably contributed to the number of fatalities registered on Ghana's roadways each year [30]. Although numerous African nations have made strides in reducing road fatalities, some have encountered challenges in this effort. Ghana, like several others, faces difficulties in effectively addressing this issue. Over the last three decades, traffic injuries and deaths in Africa have increased [31]. In 2005, South Africa, one of the most industrialized countries on the African continent, had seventeen (17) allowed automobiles per 100 citizens and no sign of a decrease in road traffic accident deaths as of now [32]. Forecasting future RTA-related deaths worldwide is difficult, although past patterns might be thought to give a realistic picture of what may occur later. However, a few nations thoroughly veer off from these expectations. Moreover, drifts in numerous parts of the world are inconsistent, and there is a confirmation of an increment in deaths in Africa and Asia/Pacific. Statistics from developing nations are consistent with changes in the total number of road traffic accidents recorded year after year. Annually, an estimated 1.2 million individuals succumb to fatalities resulting from RTAs, and another fifty (50) million are injured. Statistical analysts have forecasted that these descriptive statistics will increase by about 65% over the next 20 years if care is not taken [33], [34], [35]. 75% of road traffic deaths came about because vehicles collided with each other in low-earning income countries despite owning only 32% of yearly fatalities for every 10,000 cars around the world, making this claim unbelievable. Globally, an estimated cost of US$ 518 billion is spent on RTAs [36]. The share of the developing countries is about US $100 billion, representing 1 to 3 per cent of their gross national product [37]. These stunning numbers indicate that road traffic accidents happen on all landmasses and in every nation. Numerical and computational approaches such as those suggested by [38], [39], [40], [41], [42] can be employed as baseline mathematical models in conjunction with optimization algorithms to help reduce the alarming rate of the occurrence RTAs.

Recognizing the limitations of traditional regression techniques, particularly in handling road traffic accident-related cases due to their reliance on independence assumptions, numerous studies have shifted toward time series methodologies. Approaches such as ARMA, ARIMA, DRAG, state space models, and structural models are favoured for their ability to enhance the forecasting of factors related to RTAs. Models have additionally been utilized to examine injuries and deaths caused by RTAs. Various models have been used to model road accident data. [43] estimated the influence of speed limit modifications on the number of road crashes in metropolitan and provincial interstate thruways in the United States using a structural equation of stochastic modelling technique. [44] analyzed RTAs in Kuwait using an Autoregressive Integrated Moving Averages (Box Jenkins) model and compared it to Artificial Neural Networks (ANN) to predict RTA deaths in Kuwait. The study found that ANN was superior if there should arise an occurrence of long-term series without regular variations of accidents. Several researchers have used collision prediction models to model RTAs in various regions of the world. However, due to differences in numerous parameters in different geographical locations, it becomes challenging to apply models that have worked elsewhere in the globe to data gathered from other parts of the world [45]. In Ghana, there has been minimal statistical modelling of RTAs. This problem stems from the unavailability of data acquisition on road accident cases by the authorities in charge of road accident data. Considering the rate at which RTAs are increasing annually in Ghana, there is a need for this study. As a result, statistical analysis of the Madina-Adenta highway RTAs is required to determine the validity or falsity of current literature on RTAs in Ghana. When seasonal patterns in the road traffic accident data are validated, statistical models such as SARIMA and FB Prophet would be employed to fit a model to the RTAs data for improved prediction and decision-making. The education and research department of the National Motor Transport and Traffic Unit (MTTU) has used descriptive statistical techniques and charts for reporting road traffic accidents in Ghana over the past few years. This method's notable drawback lies in its failure to provide essential estimates of road accident occurrences, injuries, and fatalities in Ghana, hampering the ability of the National Road Safety Commission (NRSC) and Motor Transport and Traffic Unit (MTTU) stakeholders to make informed projections. Utilizing time series models like SARIMA and FB Prophet is, therefore, deemed crucial in addressing this knowledge gap.

A significant limitation to researchers in RTA research is the inability to obtain data on people who suffer from road accidents. In most parts of the world, people at an accident scene may fail to report the incident to the police for records to be taken, or if it is reported to the police, they fail to keep the records. Additionally, the emergency unit of various hospitals refuses to keep records of RTA victims once they are admitted [46]. In Ghana, accurate data on RTA cases are usually hard to come by. The information is inadequate even if acquired, mainly because not all accidents are reported to the police for records to be kept [47]. Furthermore, the police may have neglected to complete some of the accident report forms on RTAs submitted to them. However, other researchers who have utilized data on RTAs from MTTU in Ghana have provided adequate proof that their data is credible. This research makes several key contributions. Firstly, it showcases the application of the SARIMA model for capturing temporal patterns in accident data. Additionally, it introduces the implementation of the Facebook Prophet model, which adeptly handles holidays, special events, and outliers. As a result of incorporating potential changepoints into the study, the models are more capable of adapting to shifts in accident patterns than traditional methods. A rigorous comparative analysis of SARIMA and Facebook Prophet models evaluates their predictive capabilities, collectively providing an innovative and practical framework for accurate road traffic accident forecasting. Due to the increasing rate of RTAs in Ghana, undertaking this research is helpful. The results and findings of this study would be beneficial for road safety planning to help minimize road traffic accidents and fatalities in Ghana. The time series model developed in this study is recommended for use by the MTTU, NRSC, and relevant stakeholders to help monitor the efficacy of diverse road safety policies. Additionally, the study's findings will contribute to the body of academic literature concerning RTAs

The remainder of the paper is organized as follows: Section 2 discusses the data and methods used for the study, including ARMA, ARIMA, SARIMA, FB Prophet models, SARIMA model building process, model identification tools, model diagnostics, and model accuracy. Section 3 presents and discusses the results of the investigation. Section 4 concludes the research and provides recommendations.

## 2 Data and methods

Secondary RTAs data on the Madina-Adenta Highway were retrieved from police reports from 2013 to 2019 and analyzed using univariate SARIMA and FB Prophet time series model with potential changepoints. The recorded number of RTAs data used in the study include rear-end collisions, head-on collisions, side impact collisions, rollovers, pedestrian or cyclist Accidents, multi-vehicle pileups and run-off accidents. Monthly RTA data from 2013 to 2018 (72 months) were used in building the two models, while the monthly RTAs for 2019 (12 months) were used in testing the accuracy of the two models under consideration. Data from 2020 to the first half of 2023 of the number of Road Traffic Accidents (RTAs) per month were regrettably excluded from this study due to unforeseen circumstances resulting from the COVID-19 pandemic. These circumstances led to non-representative and incomplete RTA data specific to the Madina-Adenta Highway. The study focused on analyzing RTA data from this highway, revealing a conspicuous seasonal pattern. This observation prompted the application of SARIMA and FB Prophet models. The study's analysis was conducted using the R programming language. The study's data and codes are publicly accessible on GitHub via the repository located at github.com/Agyemang1z/Road-Accidents.

### 2.1 AutoRegressive moving average (ARMA) model

The autoregressive moving average ARMA (p,q) model is formulated by the combination of autoregressive AR (*p*) and moving average MA (*q*) model, which is a suitable model for univariate time series data. The AR (*p*) model is given mathematically by (1):

(1) $$x_{t}=\vartheta_{0}+\vartheta_{1}x_{t-1}+\;\vartheta_{2}x_{t-2}+.\;\;.\;\;.\;+\vartheta_{p}x_{t-p}+\;\varepsilon_{t}=\vartheta_{0}+\sum_{i=1}^{p}\vartheta_{i}x_{t-i}+\;\varepsilon_{t}$$

where $x_{t}$ are the observed values, $\varepsilon_{t}$ is random shocks at time *t*, $\vartheta_{i}\;\left(i=1\;,\;2\;,\;\;\;.\;\;.\;\;.\;\;,\;\;k\right)$ are the parameters of the AR(p) model, $\vartheta_{0}$ is the constant term, and *p* is the order of the time series model.

The MA(q) model is likewise given by (2):

(2) $$x_{t}=\;\mu +\;\varepsilon_{t}-\alpha_{1}\varepsilon_{t-1}-\alpha \varepsilon_{t-2}-\;.\;\;.\;\;.\;-\;\alpha_{q}\varepsilon_{t-q}\;=\mu +\;\varepsilon_{t}-\sum_{i=1}^{q}\alpha_{i}\varepsilon_{t-i}$$

where *μ* is the mean of the series, $\alpha_{i}\;\left(i=1\;,\;2\;,\;\;\;.\;\;.\;\;.\;\;,\;\;q\right)$ represents parameters of the model with order *q*, with random errors $\varepsilon_{t}$ are assumed as a white noise process.

The mixed autoregressive moving average ARMA(p,q) model is also expressed mathematically in (3) by:

(3) $$y_{t}=\mu +\;\sum_{i=1}^{p}\vartheta_{i}x_{t-i}+\;\varepsilon_{t}-\sum_{i=1}^{q}{\alpha_{1}}_{i}\varepsilon_{t-i}$$

where the order (p,q) represents *p* order for autoregressive AR(p) and *q* for the moving average MA(q) terms.

### 2.2 AutoRegressive integrated moving average (ARIMA) model

The ARIMA(p,d,q) model using the lag operator is mathematically expressed in (4) as:

$$\vartheta \left(L\right){\left(1-L\right)}^{d}x_{t}=\mu +\;\alpha \left(L\right)\varepsilon_{t}$$

(4) $$\left(1-\sum_{i=1}^{p}\vartheta_{i}L^{i}\right){\left(1-L\right)}^{d}x_{t}=\mu +\left(1-\sum_{i=1}^{p}\alpha_{i}L^{i}\right)\epsilon_{t}$$

The order of autoregressive, integrated, and moving average terms of the model are given respectively by *p*, *d* and *q*; *d* is the differencing required to achieve series stationarity.

### 2.3 Box-Jenkins seasonal ARIMA (SARIMA) model

Many real-world time series datasets feature a seasonal component that repeats after every *S* observation. For example, consider utilizing a monthly observation time series dataset, where S=12. We can generally anticipate that $X_{t}$ to a large extent rely on $X_{t-12}$ and probably $X_{t-24}$ in addition to terms such as $X_{t-1,\;}X_{t-2},\ldots$. The Box and Jenkins generalization ARIMA(p,d,q) include seasonal components and are often characterized as a general multiplicative Seasonal ARIMA model abbreviated as SARIMA $\left(p,d,q\right)\times {\left(P,D,Q\right)}_{S}$ model and expressed mathematically in the study in (5) by:

(5) $$\phi_{p}\left(B\right)\Phi_{P}\left(B^{s}\right)\nabla^{d}{\nabla_{S}}^{D}X_{t}=\theta_{q}\left(B\right)\Theta_{Q}\left(B^{S}\right)Z_{t}$$

Where *S* denotes the seasonal lag, *B* denotes the backshift operator and $Z_{t}$ is the random error component. $\phi_{p}$ and $\Phi_{P}$ are the non-seasonal and autoregressive seasonal parameters. Additionally, $\theta_{q}$ and $\Theta_{Q}$ are the non-seasonal and moving average seasonal parameters. *p* and *q* are, respectively, the orders of non-seasonal autoregressive and moving average parameters, whilst *P* and *Q* are orders of autoregressive and moving average seasonal parameters, respectively. Lastly, *d* and *D* respectively represent the non-seasonal and seasonal differences. $\nabla^{d}$ means we apply the ∇ operator *d* times and similarly for ${\nabla_{S}}^{D}$.

### 2.4 ARIMA model building process

The ARIMA model uses a three-stage approach to get a suitable model for a forecast. These include:

1. Model Identification: The model identification involves determining if the time series data is stationary or non-stationary [48]. If it is non-stationary, determine the degree of differencing needed to make it stationary. The acquisition of the AR order *p* and the MA order *q* follows afterwards. Typically, the non-stationary time series data is frequently shown by an autocorrelation graph with slow decay. For this study, the Augmented Dickey-Fuller Test (ADF) test was used to test for series stationarity.
2. Model Estimation: This entails determining the best feasible estimates for the Box-Jenkins model parameters [49]. Nonlinear least squares and maximum likelihood estimation are the primary methodologies for fitting Box-Jenkins models. The parameters in this study were estimated using Maximum Likelihood Estimation (MLE).
3. Model Diagnostic: This stage checks if the model is adequate or not. If the model is inadequate, it is essential to return to stage one and choose a better model. Once the model has been selected, estimated, validated, and determined to be acceptable, it is utilized to generate forecasts.

### 2.5 Test of significance of model coefficients

For each coefficient, the estimated t-value is given by (6) as:

(6) $$t=\frac{estimated\;coefficient}{standard\;error}$$

If |t|≥2, the estimated coefficient is significantly different from zero (0), and the model coefficient is statistically significant. Also, if the p-value of a model coefficient is less than the 5% significance level, the estimated coefficient is adjudged statistically substantial and otherwise.

### 2.6 Model identification tools

They evaluate the balance between model adequacy and model complexity. Various indicators measuring the quality of fit applied in this study's model identification process include Akaike Information Criterion (AIC), corrected Akaike Information Criterion (AICc), Bayesian Information Criterion (BIC), Mean Absolute Percentage Error (MAPE), Mean Square Error (MSE), Root Mean Square Error (RMSE), and Mean Absolute Error (MAE). The AIC uses the MLE approach. The MLE technique is utilized to estimate a variety of feasible SARIMA models for this approach, and each AIC computed using (7)

(7) AIC=−2ln⁡L+2W

where ln⁡L is the model's log-likelihood, and *W* is the number of model parameters. In the case of two or more competing models, the one with the lower AIC is superior. The AIC exhibits bias, particularly evident when the ratio of parameters to available data is high. [50] demonstrated that the tendency might be approximated by introducing an additional non-static penalty factor to the AIC, resulting in the development of the corrected AIC, denoted by AICc, and mathematically given by (8) as

(8) $$AIC_{c}=AIC+\frac{2W\left(W+1\right)}{N-W-1}$$

where *N* is the sample size or the number of time series observations.

The BIC, like AIC, also uses the MLE. It is expressed by (9) as:

(9) BIC=−2ln⁡L+Wln⁡(N)

The BIC penalizes the number of estimated model parameters more severely than the AIC. Applying minimal BIC for model selection results in a model with fewer parameters than that chosen for AIC. According to the concept of parsimony, BIC is considerably superior in model selection over AIC. A lower BIC value indicates that the model fits better.

### 2.7 Test of model diagnostics for SARIMA model

The Box-Pierce and Ljung-Box tests is employed to check the adequacy of the study's estimated model. The Ljung-Box test fits residual (error term) randomness based on several lags. If the autocorrelations of the residuals are small, the model does not exhibit a significant lack of fit and is thus assumed adequate. The Lilliefors (KS) test is also used in this study to check for the normality of the model's residuals, and it must have a p-value more significant than 0.05; otherwise, the model's residuals are considered not to be normally distributed. The Ljung-Box statistics is a function of the accumulated sample autocorrelation, $\rho_{h}$, up to any specified time lag *k*. It is obtained as a function of *h* given by (10) as

(10) $$Q\;=\;n\left(n+2\right)\sum_{h=1}^{k}\frac{\rho_{h}^{2}}{n-h}$$

where $Q∼\chi_{\alpha ,n-p-q}^{2}$, and *n* is the number of data points that can be used after any differencing processes. When the calculated value of *Q* is obtained, the critical region for rejection of the hypothesis of randomness is $Q>\chi_{\alpha ,n-p-q}^{2}$. This means that the model under consideration is inadequate but adequate if otherwise. When the model is insufficient, there arises a need to fit an appropriate model. That is, going back to the model identification and developing a better model.

### 2.8 Test of model accuracy

Detecting the best-fit model based on accuracy ensures that the chosen model is not over fitted. It is important to note that a high error rate indicates that the model is built poorly, whereas a low error rate indicates that it is built well. The accuracy of the two competitive models were computed using (11), (12), (13), (14) and (15) respectively: MAPE, MAE(MAD), *MSE*, RMSE and Theil U1 Statistic (*τ*).

(11) $$MAPE=\frac{1}{n}\sum_{t=1}^{n}\frac{\left|y_{t}-{\overset{ˆ}{y}}_{t}\right|}{y_{t}}\times 100\text{\%}.$$

(12) $$MAE(MAD)=\frac{1}{n}\sum_{t=1}^{n}|y_{t}-{\overset{ˆ}{y}}_{t}|.$$

(13) $$MSE=\frac{\sum_{t=1}^{n}{\left(y_{t}-{\overset{ˆ}{y}}_{t}\right)}^{2}}{n}.$$

(14) $$RMSE=\sqrt{\frac{\sum_{t=1}^{n}{\left(y_{t}-{\overset{ˆ}{y}}_{t}\right)}^{2}}{n}}.$$

(15) $$\tau =\sqrt{\frac{1}{n}\sum_{t=1}^{n}\epsilon_{t}^{2}}÷\left(\sqrt{\frac{1}{n}\sum_{t=1}^{n}y_{t}^{2}}+\sqrt{\frac{1}{n}\sum_{t=1}^{n}{\overset{ˆ}{y}}_{t}^{2}}\right),.$$

where $y_{t}$ are the actual values, ${\overset{ˆ}{y}}_{t}$ are the forecast values and $y_{t}-{\overset{ˆ}{y}}_{t}=\epsilon_{t}$ are the forecast errors. 0≤τ≤1, for τ≊0 implies good fit of model to data and τ≊0 implies poor fit of model to data.

### 2.9 Forecasting

After successfully identifying, estimating, diagnosing, and deciding on the appropriate time series model to use, forecasting can be done. If the current time is denoted by *t*, the forecast for $Y_{t+r}$ is the *r*− period ahead forecast and denoted by ${\overset{ˆ}{Y}}_{t+r}$. The infinite MA representation of the forecast is given in (16) by;

(16) $${\overset{ˆ}{Y}}_{t+r}=\mu +\sum_{i=1}^{\infty }\psi_{i}\varepsilon_{t+r-i}$$

and an ARIMA(p,d,q) process at time t+r (that is, a period in the future) is given in (17):

(17) $${\overset{ˆ}{Y}}_{t+r}=\sum_{i=1}^{p+d}\emptyset_{i}y_{t+r-i}+\varepsilon_{t+r}-\;\sum_{i=1}^{q}\theta_{i}\varepsilon_{t+r-i}$$

where, $\psi_{i}$ is the weight (a constant). Once a forecast is obtained for $Y_{t+1}$, it can be used to obtain a forecast for $Y_{t+2}$ and then, these two generate a forecast for $Y_{t+3}$. This can be used to acquire forecasts for any point in time.

### 2.10 Facebook Prophet forecasting model

Developed by Facebook, the FB Prophet, an additive regression model is in high demand for forecasting purposes due to its three main features: trend, seasonality, and holiday. The model is expressed in (18) as

(18) y(t)=α(t)+β(t)+η(t)+ε(t)

where y(t) is the forecast; the model parameters α(t), β(t) and η(t) are respectively the trend (non-periodic changes), seasonal (periodic changes) and holidays effects, which gives irregular schedules. ε(t) is the error term of the forecast y(t) which represent any unusual changes. The FB Prophet model adopts a Fourier series to fit models with seasonality effects s(t) represented in (19) as

(19) $$s\left(t\right)=\sum_{k=1}^{N}\alpha_{k}\cos\left(\frac{2\pi kt}{p}\right)+\beta_{k}\sin\left(\frac{2\pi kt}{p}\right)$$

where *p* is the period of the seasonal pattern, $\alpha_{k}$ and $\beta_{k}$ are the Fourier coefficients. Employing the data's rising points as a reference, the Prophet model adopts a logistic growth curve trend to discern trends. FB Prophet is adept at managing time series data characterized by significant seasonal fluctuations and a substantial historical data span. Notably, the Prophet model effectively manages outliers, even in scenarios involving missing data or shifts in trends [51], [52]. The effective application of a Prophet model necessitates the variables y (target) and ds (Date Time) in the time series. It demonstrates optimal performance when applied to datasets encompassing multiple seasons and featuring notable seasonal impacts [53]. For the purpose of this study, the potential change points were chosen as the months with the major holidays in Ghana. This study chose January, March, April, May and December as our potential changepoints and the number of changepoints was set as 30. We operationalized the trend model using a saturating growth approach, establishing the logistic growth model's carrying capacity at 10. We set the interval width and change point prior Scale to 0.8 and 0.05 respectively.

The introduction and comparison of the FB Prophet model (with potential changepoints) with other competitive time series models (such as SARIMA) to forecast RTAs in Ghana has not been explored and to the best of our knowledge, this is the first study to explore the FB Prophet model in this domain. Figure 1, Figure 2 presents the working model of the SARIMA and FB Prophet adopted for the study.

**Figure 1:** Working model of ARIMA adopted from [53].

**Figure 2:** Working model of Facebook Prophet adopted from [53].

### 2.11 Comparison between Facebook Prophet and ARIMA models

1. Model Complexity: Facebook Prophet has been designed to be a user-friendly forecasting tool with minimal configuration requirements [54]. It automates several steps involved in time series forecasting, such as handling seasonality, trend detection, and outliers. ARIMA is a more traditional and widely used time series forecasting model. A key aspect of ARIMA models is tuning model parameters, such as order (p,d,q) values for autoregressive, differencing, and moving average components.
2. Seasonality Handling: As part of its integrated functionality, FB Prophet is able to handle a variety of seasonalities, such as daily, weekly, and yearly patterns [55]. It can handle multiple seasonal components and also handle irregular holidays and events. Models that use ARIMA can also handle seasonal data through seasonal differencing or by manually incorporating seasonal components.
3. Trend Detection and Outlier handling: FB Prophet automatically detects and models both linear and non-linear trends and can handle outliers in the data. It can identify and adjust for these outliers, preventing them from overly influencing the forecast and can handle situations where the trend changes over time. ARIMA models can capture linear trends but may not handle non-linear trends effectively.
4. Interpretability: The FB Prophet provides a more interpretable forecast due to its breakdown into the trend, seasonality, and holiday components. In addition, it provides visualizations and diagnostics for evaluating the model's performance. The ARIMA model is less interpretable since it focuses mostly on the statistical properties of the time series. An understanding of the underlying mathematics is necessary to interpret the model parameters and diagnostics of an ARIMA model.

### 2.12 Examples of solving optimization problems in road traffic accident research

It is worth knowing that solving optimization problems in road accident research is key to reducing toad traffic accidents. Below are three concrete examples of solving optimization problems in road accident related research.

1. Traffic Signal Timing Optimization
  • Problem: Enhancing the synchronization of traffic signals at intersections to alleviate congestion and lower the probability of accidents.
  • Solution: By optimizing the timing of traffic signals, researchers and traffic engineers can work to minimize the likelihood of accidents occurring. An objective function is defined, which could include minimizing the total number of conflict points (locations where accidents are more likely to occur) or maximizing the throughput of vehicles. Constraints are established to ensure that traffic signal timings adhere to safety and operational standards. These constraints may include minimum green time, maximum cycle length, and pedestrian crossing times. Various optimization algorithms, such as those established by [56], [57] may be applied to find the optimal signal timing plan that minimizes the objective function while satisfying the constraints. The optimized signal timing plan is then simulated to assess its impact on traffic flow and safety. Once an optimized signal timing plan is validated, it can be implemented at the intersection.
2. Route Planning for Emergency Services
  • Problem: Finding the optimal routes for emergency vehicles (e.g., ambulances, fire trucks) to reach accident scenes quickly while avoiding traffic congestion.
  • Solution: Applying optimization algorithms such as that established by [58], [59], [60] to take into account real-time traffic data, accident locations, and the urgency of the situation. These algorithms can recommend the fastest and safest routes for emergency responders, potentially saving lives by reducing response times.
3. Vehicle Fleet Optimization for Safety Inspections
  • Problem: Optimizing the scheduling and routing of safety inspection teams to inspect a large number of vehicles efficiently, ensuring compliance with safety regulations and reducing the risk of accidents due to faulty vehicles.
  • Solution: Use vehicle routing optimization algorithms to determine the best inspection routes for a fleet of inspectors, considering factors like the locations of inspection sites, inspection durations, and traffic conditions. The goal is to maximize the number of inspections performed within a given time frame while minimizing travel distance and time.

These examples demonstrate how optimization techniques can be applied in road traffic accident research to enhance safety, improve traffic flow, and allocate resources effectively. They leverage data and modelling to make informed decisions and reduce the risk of accidents on the road.

## 3 Results and discussion

This section presents the outcomes of the forecast generated by the SARIMA and FB Prophet models.

Over the seven-year span under study, January demonstrated the lowest occurrence of road accidents, with an average of 29 incidents. The first and third quarters each witnessed an average of 33 road accidents per month. Notably, the fourth quarter experienced the highest monthly average of reported RTAs, with an average of 37 incidents, marking this period as the most perilous for drivers, passengers, pedestrians, and other road users. Unexpectedly, the most perilous month of the year is November, despite the festive activities typically associated with December in Ghana. November falls within the fourth quarter and records an average of 41 traffic accidents per month. The ratio between the highest average value (November) and the lowest average value (January) stands at 41.38%. The standard deviations of the monthly road accidents cases depicted in Fig. 3 by year are: 10 (2013), 11 (2014), 8 (2015), 4 (2016), 11 (2017), 12 (2018), and 4 (2019).

**Figure 3:** Box-plot with data on traffic accidents by months (2013–2019).

### 3.1 Development of the SARIMA model

Fig. 4 depicts the frequency of RTAs on the Madina-Adenta highway as spikes and troughs increase and decrease. The average number of traffic accidents per year are 26 (2013), 35 (2014), 27 (2015), 29 (2016), 39 (2017), 41 (2018) and 42 (2019). From the reference year 2013, it is evident that the average number of road accidents has risen by 34.62% (2014), 3.85% (2015), 11.54% (2016), 50.00% (2017), 57.69% (2018) and 61.54% (2019). From Fig. 4, we observe some upward and downward surges in the series. Also, Fig. 4 shows that the monthly RTAs time series dataset under examination has a solid and persistent seasonal tendency. This indicates that seasonal components exist in the monthly RTAs. This further suggests that the monthly RTAs data on the Madina-Adenta highway is non-stationary. To effectively apply an appropriate time series model to the RTA data, it's imperative to eliminate both the seasonality and trend present within the dataset. The single exponential smoothing method was employed to deal with the seasonality and trend components as suggested by the  function in R.

**Figure 4:** Time series plot of Road Traffic Accident cases from 2013 to 2019.

### 3.2 Single exponential smoothing method

The road traffic accident data underwent a first-order differencing method to effectively eliminate both the trend and seasonality from the original dataset. Fig. 5 helps us to see that the differenced data exhibits stationarity with constant mean and variance. The Augmented Dickey-Fuller Test (ADF) test was employed to confirm series stationarity test.

**Figure 5:** Single Exponential plot of Road Traffic Accident cases.

We reject the null hypothesis of non-stationarity and conclude that the first differenced RTAs data is stationary since 0.0100 < 0.05 as evident in Table 1.

**Table 1:** ADF test for Level Stationarity.

Test	Statistic	Lag Order	P-value
ADF	−5.8053	4	0.0100

### 3.3 Autocorrelation and partial autocorrelation function plots of the first difference

From Fig. 6(a), looking at the autocorrelation function with the error limits, autocorrelation at lag one is significant. This depicts a possible behaviour of MA (1). For the plot of ACF, we notice sinusoidal waves shown in the autocorrelation plot.

**Figure 6:** Plot of the ACF and PACF of First Difference road traffic accident cases.

Fig. 6(b) depicts the partial autocorrelation function plot, which demonstrates that the partial autocorrelation coefficient exceeds the error bounds at lags 1, 2, and 4, which are significant. The error limit at lag 3 is insignificant, and it is the first to do so. Since the PACF cuts off after lags 1, 2 and lag 4, this suggests possible behaviour of SMA (1), SMA (2) or SMA (4). The ACF and PACF plots suggest that Q=1,2or4, p=1,P=1, d=1,D=0 and q=1 would be needed to model the road traffic accident data. The following tentative models; $SARIMA\;\left(1,1,1\right)\times {\left(1,0,1\right)}_{12}$, $SARIMA\;\left(1,1,1\right)\times {\left(1,0,0\right)}_{12}$, $SARIMA\;\left(1,1,0\right)\times {\left(0,0,1\right)}_{12}$, $SARIMA\;\left(0,1,1\right)\times {\left(1,0,0\right)}_{12}$, $SARIMA\;\left(0,1,2\right)\times {\left(1,0,0\right)}_{12}$, $SARIMA\;\left(1,1,2\right)\times {\left(1,0,0\right)}_{12}$ and $SARIMA\;\left(0,1,3\right)\times {\left(1,0,2\right)}_{12}$ can be suggested after careful examination of the ACF and PACF plots in Fig. 6.

### 3.4 Possible seasonal ARIMA models parameter estimation

The tables below display the final parameter estimates of the possible seasonal ARIMA models under consideration with their respective coefficients, standard error, and p-values.

From Table 2, AR(1), MA (1) and SMA (1) are statistically significant at the 5% significance level.

**Table 2:** Final parameter estimates of $SARIMA\;\left(1,1,1\right)\times {\left(1,0,1\right)}_{12}$.

Parameter	Coefficient	Standard Error	Z-value	P-value
AR (1)	−0.0057	0.0007	−7.8014	0.000^⁎⁎⁎^
MA (1)	−0.7831	0.0069	−1111.2357	0.000^⁎⁎⁎^
SAR (1)	−0.5513	NaN	NaN	NaN
SMA (1)	0.3654	0.0028	132.0225	0.000^⁎⁎⁎^

From Table 3, MA (1) with a coefficient of -0.8080 and a Z-value of -8.2895 is statistically significant.

**Table 3:** Final parameter estimates of $SARIMA\;\left(1,1,1\right)\times {\left(1,0,0\right)}_{12}$.

Parameter	Coefficient	Standard Error	Z-value	P-value
AR (1)	0.0422	0.1543	0.2733	0.7846
MA (1)	−0.8080	0.0975	−8.2895	0.000^⁎⁎⁎^
SAR (1)	−0.2176	0.1363	−1.5965	0.1104

AR (1) with a coefficient of -0.4929 and a standard error of 0.1075 statistically significant as seen in Table 4.

**Table 4:** Final parameter estimates of $SARIMA\;\left(1,1,0\right)\times {\left(0,0,1\right)}_{12}$.

Parameter	Coefficient	Standard Error	Z-value	P-value
AR (1)	−0.4929	0.1075	−4.5863	0.000^⁎⁎⁎^
SMA (1)	−0.1678	0.1325	−1.2654	0.2057

From Table 5, MA (1) is statistically significant with p-value <0.05.

**Table 5:** Final parameter estimates of $SARIMA\;\left(0,1,1\right)\times {\left(1,0,0\right)}_{12}$.

Parameter	Coefficient	Standard Error	Z-value	P-value
MA (1)	−0.7905	0.0807	−9.7978	0.000^⁎⁎⁎^
SAR (1)	−0.2170	0.1364	−1.5911	0.1116

From Table 6, MA (1) is statistically significant with p-value <0.05.

**Table 6:** Final parameter estimates of $SARIMA\;\left(0,1,2\right)\times {\left(1,0,0\right)}_{12}$.

Parameter	Coefficient	Standard Error	Z-value	P-value
MA (1)	−0.7665	0.1186	−6.4636	0.000^⁎⁎⁎^
MA (2)	−0.0325	0.1209	−0.2686	0.7883
SAR (1)	−0.2179	0.1363	−1.5983	0.1100

From Table 7, MA (1) is also statistically significant at alpha level of <0.05.

**Table 7:** Final parameter estimates of $SARIMA\;\left(1,1,1\right)\times {\left(1,0,0\right)}_{12}$.

Parameter	Coefficient	Standard Error	Z-value	P-value
AR (1)	0.0422	0.1543	0.2733	0.7846
MA (1)	−0.8080	0.0975	−8.2895	0.000^⁎⁎⁎^
SAR (1)	−0.2176	0.1363	−1.5965	0.1104

MA(1) is also statistically significant in the $SARIMA\;\left(0,1,3\right)\times {\left(1,0,2\right)}_{12}$ model as seen in Table 8.

**Table 8:** Final parameter estimates of $SARIMA\;\left(0,1,3\right)\times {\left(1,0,2\right)}_{12}$.

Parameter	Coefficient	Standard Error	Z-value	P-value
MA (1)	−0.7654	0.1204	−6.3592	0.000^⁎⁎⁎^
MA (2)	−0.0072	0.1710	−0.0420	0.9665
MA (3)	−0.0269	0.1639	−0.1645	0.8693
SAR (1)	−0.3745	0.4348	−0.8615	0.3890
SMA (1)	0.1952	0.4297	0.4543	0.6496
SMA (2)	0.1129	0.2598	0.4346	0.6638

### 3.5 Fitting the suitable SARIMA model to road accident time series data

Both the initial differenced ACF and PACF plots were rigorously examined when modelling the road traffic accident series data to produce the suitable-fitted model based on their respective *AIC*, $AIC_{C}$ and *BIC* values.

From Table 9, comparing the *AIC*, $AIC_{C}$ and *BIC* values of the candidate models, it can be deduced that the SARIMA $\left(1,1,0\right)\times {\left(0,0,1\right)}_{12}$ (highlighted in red) has an *AIC* value of 538.56, an $AIC_{C}$ value of 538.92 and a *BIC* value of 545.35 which are the lowest accuracies of all the tentative SARIMA models constructed. Therefore, per the model selection criteria, SARIMA $\left(1,1,0\right)\times {\left(0,0,1\right)}_{12}$ is the suitable SARIMA time series model for modelling the Madina-Adenta highway road traffic accident.

**Table 9:** Potential SARIMA models with their *AIC*, *AIC*_*C*_ and *BIC* values.

The general multiplicative Seasonal ARIMA model is thus given in the study by equation (5) as:

$$\phi_{p}\left(B\right)\Phi_{P}\left(B^{s}\right)\nabla^{d}{\nabla_{S}}^{D}X_{t}=\theta_{q}\left(B\right)\Theta_{Q}\left(B^{S}\right)Z_{t}$$

Hence, the seasonal ARIMA (0,1,1)×(1,0,0) can be represented in (20) as

(20) $$\phi_{0}\left(B\right)\Phi_{1}\left(B^{12}\right)\nabla^{1}{\nabla_{12}}^{0}X_{t}=\theta_{0}\left(B\right)\Theta_{0}\left(B^{12}\right)Z_{t}$$

### 3.6 Diagnostic checking of estimated model

The suitable-fitted model for modelling the road accident data is then tested further to make theoretical conclusions about the model as a good fit and an optimal model for both estimation and forecasting.

From Table 10, Given the p-value of 0.8864, which exceeds the significance threshold of 0.05, we conclude that the residuals of the estimated model demonstrate independence and follow an identically distributed or white noise process. Hence, the model displays no substantial lack of fit.

**Table 10:** Ljung-Box test of SARIMA $\left(0,1,1\right)\times {\left(1,0,0\right)}_{12}$.

Test	Statistic	P-value
Ljung-Box	6.5417	0.8864

At a 5% significance level, since the p-value is greater than the alpha level (thus, 0.2364 > 0.05), the residuals of the estimated SARIMA $\left(0,1,1\right)\times {\left(1,0,0\right)}_{12}$ model are normally distributed as evident in Table 11.

**Table 11:** Lilliefors (KS) Normality test of SARIMA $\left(0,1,1\right)\times {\left(1,0,0\right)}_{12}$.

Test	Statistic	P-value
Lilliefors (KS)	0.0841	0.2364

### 3.7 Test of model adequacy of SARIMA

The limits of the 2*σ* are given by $\pm Z_{\frac{\alpha }{2}}\times \frac{1}{\sqrt{n}}$.

$$-1.96\left(\frac{1}{\sqrt{72}}\right)\leq r\leq 1.96\left(\frac{1}{\sqrt{72}}\right)$$

This is simplified as −0.2310≤r≤0.2310. Hence, the confidence interval of the random error spans across two (2) standard deviations. Fig. 7 shows two blue horizontal lines indicating this claim. It could be seen that the errors are within ±0.2310 as evident in the ACF/PACF plots. It should also be noted that the plot of these autocorrelations shows no systematic structure, indicating that the residuals are purely random.

**Figure 7:** Plot of ACF and PACF plot of residuals of SARIMA $\left(0,1,1\right)\times {\left(1,0,0\right)}_{12}$ model.

### 3.8 Box-Pierce test for larger lags

The modified Ljung-Box test (Box-Pierce test) for larger lags was employed to ascertain whether the proposed model is adequate for forecasting.

Observing Table 12, it is apparent that the p-values at different lags considerably surpass the 0.05 significance level. As a result, we lack substantial evidence to reject our model. Given its adequacy for lags 12, 24, 36, 48, and 60, it is plausible to assume its adequacy for larger lags as well. Hence, the SARIMA $\left(0,1,1\right)\times {\left(1,0,0\right)}_{12}$ model is adequate at a 0.05 level of significance and can be used to forecast future road accident cases optimally.

**Table 12:** Modified Ljung-Box (Box-Pierce test) for larger lags of SARIMA $\left(0,1,1\right)\times {\left(1,0,0\right)}_{12}$.

Lags	Chi-Square Statistic	P-value
12	5.7045	0.9302
24	8.1798	0.9989
36	14.956	0.9992
48	19.566	0.9999
60	25.717	1.0000

### 3.9 Evaluation of SARIMA model

It is clear from Table 13 that the SARIMA $\left(0,1,1\right)\times {\left(1,0,0\right)}_{12}$ model developed for RTAs on the Madina-Adenta Highway has a forecast accuracy of 93.1025%, displayed by the model's MAPE of 6.8975% which is indicative of highly accurate forecasting as suggested by [61]. A *τ* statistic of 0.0376 further indicates good model fit.

**Table 13:** Out of sample Validation for $SARIMA\;\left(0,1,1\right)\times {\left(1,0,0\right)}_{12}$ with Forecast Performance Statistics.

Month Year	*y*_*t*_	${\overset{ˆ}{y}}_{t}$	$y_{t}^{2}$	${\overset{ˆ}{y}}_{t}^{2}$	*ϵ*_*t*_	|*ϵ*_*t*_|	$\epsilon_{t}^{2}$	$\left|\frac{\epsilon_{t}}{y_{t}}\right|$	|% *Error*|
Jan 2019	38	43	1444	1849	5	5	25	0.1316	13.16
Feb 2019	43	47	1849	2209	4	4	16	0.0930	9.30
Mar 2019	36	40	1296	1600	4	4	16	0.1111	11.11
Apr 2019	45	44	2025	1936	−1	1	1	0.0227	2.27
May 2019	40	42	1600	1764	2	2	4	0.0500	5.00
Jun 2019	39	40	1521	1600	1	1	1	0.0256	2.56
Jul 2019	50	46	2500	2116	−4	4	16	0.0800	8.00
Aug 2019	42	43	1764	1849	1	1	1	0.0233	2.33
Sep 2019	39	44	1521	1936	5	5	25	0.1282	12.82
Oct 2019	44	42	1936	1764	−2	2	4	0.0454	4.54
Nov 2019	41	38	1681	1444	−3	3	9	0.0732	7.32
Dec 2019	46	44	2116	1936	−2	2	4	0.0435	4.35
**Total**	**503**	**513**	**21253**	**22003**		**34**	**122**	**0.8277**	

MAE	2.8333								
MAPE	6.8975								
MSE	10.1667								
RMSE	3.1885								
Theil's U1 Statistic (*τ*)	0.0376								

From Table 14, it is evident that the best model by the auto.arima function in R programming software confirms that our selected model (ARIMA(0,1,1)(1,0,0)[12]) using the diagnostic of the ACF and PACF plots is the ideal seasonal model to forecast the underlying RTAs data.

**Table 14:** Possible tentative ARIMA models extracted by auto.arima function.

Model	Evaluation Statistic
ARIMA(0,1,0)(0,0,1)[12]	569.2443
ARIMA(0,1,0)(0,0,1)[12] with drift	571.4203
ARIMA(0,1,0)(0,0,2)[12]	570.8983
ARIMA(0,1,0)(0,0,2)[12] with drift	573.145
ARIMA(0,1,0)(1,0,0)[12]	568.8583
ARIMA(0,1,0)(1,0,0)[12] with drift	571.0352
ARIMA(0,1,0)(1,0,1)[12]	570.9207
ARIMA(0,1,0)(1,0,1)[12] with drift	573.1644
ARIMA(0,1,0)(1,0,2)[12]	572.3704
ARIMA(0,1,0)(2,0,0)[12] with drift	573.0677
ARIMA(0,1,0)(2,0,1)[12]	573.0674
ARIMA(0,1,0)(2,0,1)[12] with drift	575.3814
ARIMA(0,1,0)(2,0,2)[12]	Inf
ARIMA(0,1,0)(2,0,2)[12] with drift	Inf
ARIMA(0,1,1)(0,0,1)[12] with drift	540.1289
ARIMA(0,1,1)(0,0,2)[12]	541.2295
ARIMA(0,1,1)(0,0,2)[12] with drift	542.4327
**ARIMA(0,1,1)(1,0,0)[12]**	**538.9229**
**ARIMA(0,1,1)(1,0,0)[12] with drift**	**539.9962**
ARIMA(0,1,1)(1,0,1)[12]	540.9437
ARIMA(0,1,3)(0,0,1)[12]	543.619
ARIMA(0,1,3)(0,0,1)[12] with drift	544.4773
ARIMA(0,1,3)(0,0,2)[12]	545.7991
ARIMA(1,1,1)(0,0,1)[12]	541.3203
ARIMA(1,1,1)(0,0,1)[12] with drift	542.2117
ARIMA(1,1,1)(0,0,2)[12]	543.4696
ARIMA(1,1,1)(0,0,2)[12] with drift	544.597
ARIMA(1,1,1)(1,0,0)[12]	541.0963
ARIMA(1,1,1)(1,0,0)[12] with drift	542.1079
ARIMA(1,1,1)(1,0,1)[12]	Inf
ARIMA(1,1,1)(1,0,1)[12] with drift	Inf
ARIMA(1,1,1)(1,0,2)[12]	545.4409
ARIMA(1,1,1)(1,0,2)[12] with drift	546.8489
ARIMA(1,1,1)(2,0,0)[12]	Inf
ARIMA(1,1,1)(2,0,0)[12] with drift	Inf
ARIMA(2,1,1)(0,0,1)[12]	543.6271
ARIMA(2,1,1)(0,0,1)[12] with drift	544.5017
ARIMA(2,1,1)(0,0,2)[12]	545.8267
ARIMA(2,1,1)(0,0,2)[12] with drift	546.9558
ARIMA(2,1,1)(1,0,0)[12]	543.4051
ARIMA(3,1,0)(0,0,1)[12]	549.7264
ARIMA(3,1,0)(0,0,1)[12] with drift	551.9101
ARIMA(3,1,0)(0,0,2)[12]	552.022
ARIMA(3,1,0)(0,0,2)[12] with drift	554.3071
ARIMA(3,1,0)(1,0,0)[12]	549.4729
ARIMA(4,1,0)(0,0,1)[12]	543.9409
ARIMA(4,1,0)(0,0,1)[12] with drift	546.0397
ARIMA(4,1,0)(1,0,0)[12]	543.4893
ARIMA(4,1,0)(1,0,0)[12] with drift	545.5827
ARIMA(4,1,1) with drift	548.1061
ARIMA(5,1,0) with drift	548.3584

Best model: ARIMA(0,1,1)(1,0,0)[12].

### 3.10 Evaluation of Facebook Prophet model

The performance of the FB Prophet model, with change points being the months with the major holidays in Ghana is assessed. January, March, April, May and December were chosen as potential change points.

It is evident from Table 15 and Fig. 8 that the Facebook Prophet model developed for RTAs on the Madina-Adenta Highway has a forecast accuracy of 84.3569%, displayed by the model's MAPE of 15.6431%.

**Table 15:** Out of sample Validation for Facebook Prophet model with Forecast Performance Statistics.

Month Year	*y*_*t*_	${\overset{ˆ}{y}}_{t}$	$y_{t}^{2}$	${\overset{ˆ}{y}}_{t}^{2}$	*ϵ*_*t*_	|*ϵ*_*t*_|	$\epsilon_{t}^{2}$	$\left|\frac{\epsilon_{t}}{y_{t}}\right|$	|% *Error*|
Jan 2019	38	38	1444	1444	0	0	0	0.0000	0.00
Feb 2019	43	43	0	0	0	0	0	0.0000	0.00
Mar 2019	36	55	1296	3025	−19	19	361	0.5278	52.78
Apr 2019	45	35	2025	1225	10	10	100	0.2222	22.22
May 2019	40	33	1600	1089	7	7	49	0.1750	17.50
Jun 2019	39	41	1521	1681	−2	2	4	0.0513	5.13
Jul 2019	50	38	2500	1444	12	12	144	0.2400	24.00
Aug 2019	42	42	0	0	0	0	0	0.0000	0.00
Sep 2019	39	37	1521	1369	2	2	4	0.0513	5.13
Oct 2019	44	46	1936	2116	−2	2	4	0.0455	4.54
Nov 2019	41	57	1681	3249	−16	16	256	0.3902	39.02
Dec 2019	46	38	2116	1444	8	8	64	0.1739	17.39
**Total**	**503**	**503**	**21253**	**21699**		**78**	**986**	**1.8772**	

MAE	6.5000								
MAPE	15.6431								
MSE	82.1667								
RMSE	9.0646								
Theil's U1 Statistic	0.1071

**Figure 8:** Plot of Forecasted values of Facebook Prophet model with 95% confidence limits.

The SARIMA $\left(0,1,1\right)\times {\left(1,0,0\right)}_{12}$ model developed in this study outperforms the Facebook Prophet model per their respective forecast performance statistics. It is then ideal to use the SARIMA model to make forecasts.

It is observed that road accidents on the Madina-Adenta Highway will show decreasing and increasing spikes from the start of January 2019 to the last quarter of 2019. There will be an anticipated steady pattern in RTA cases from the first quarter of 2020 and afterwards, as depicted by Fig. 9.

**Figure 9:** Plot of Forecasted values of $\left(0,1,1\right)\times {\left(1,0,0\right)}_{12}$ model with 95% confidence limits.

## 4 Conclusion and recommendation

Introducing and producing several vehicles has led to increased traffic accidents and negative consequences. Therefore, constantly reviewing, analyzing, and evaluating the existing situation is necessary. This will help identify the main causes of accidents and the most effective prevention strategies. Creating awareness campaigns to educate people on safe driving practices is also imperative. An integral facet of traffic management within a jurisdiction involves forecasting the frequency of RTAs during specific periods of the year [61]. This is mainly to get citizens informed about road safety status to understand the issue better, improve their attitudes, and improve their driving habits. Our primary objective for this study is to compare how well SARIMA and Facebook Prophet models with potential change points handle time series data with seasonal components. The study aimed to identify a suitable model that fits the Madina-Adenta RTA data and use it to forecast. The time series plot of the RTA data showed both increasing and decreasing spikes with sharp upward and downward surges, indicative of seasonality in the data. This gives a suspicion of the data being non-stationary. The RTA data was then differenced once to make it stationary. An estimated seasonal ARIMA and FB Prophet models were developed using the monthly RTA time series data from 2013 to 2018 (72 months) as the training set. The monthly RTA time series data for 2019 (12 months) were used to test the accuracy of candidate models. A comparison of all the possible model accuracy metrics (*AIC*, $AIC_{C}$ and *BIC*) of the suggested tentative models for the Madina-Adenta monthly RTAs time series data revealed that $SARIMA\;\left(0,1,1\right)\times {\left(1,0,0\right)}_{12}$ which has an *AIC* value of 538.56, $AIC_{C}$ value of 538.92 and a *BIC* value of 545.35, which were respectively the lowest among all the possible SARIMA models formulated was chosen as the suitable model in modelling the RTAs on the Madina-Adenta highway, Ghana per the selection criteria approaches. $SARIMA\;\left(0,1,1\right)\times {\left(1,0,0\right)}_{12}$ was then subjected to model diagnostic tests. The diagnostic test was conducted on the normality of the residuals, independence of the residuals and the test for model accuracy. The Lilliefors test for normality proved that the residuals were normally distributed. In contrast, the Ljung-Box test shows that the residuals were free of serial or autocorrelation and followed a white noise process. The modified Ljung-Box, also known as the Box-Pierce test for larger lags, proved significant at the 5% significance level for lags 12, 24, 36, 48 and 60, which indicates that it will be significant for larger lags, too, making the estimated model considered ideal for forecasting. A comparative analysis was then made between $SARIMA\;\left(0,1,1\right)\times {\left(1,0,0\right)}_{12}$ and FB Prophet model, where the former provided a high forecast accuracy of 93.1025% relative to the latter's forecast accuracy of 84.3569%. A Theil U1 statistic of 0.0376 for the SARIMA model compared to 0.1071 for the FB Prophet model further indicates a good model fit of the SARIMA model to the RTA data. Even though the FB Prophet model has outperformed SARIMA models in most domains regarding RTA modelling, its applicability to the Ghanaian setting is missing in action. For example, forecasting daily time series of passenger demand for urban rail transit [62], road traffic injury prediction in Northeast China [63], road traffic forecasting in Bangladesh [64]. The study, therefore, recommended that the MTTU and National Safety Road Commission (NRSC) should adopt $SARIMA\;\left(0,1,1\right)\times {\left(1,0,0\right)}_{12}$ model in their RTAs safety intervention planning activities due to its high forecast accuracy. Several avenues for further research can be pursued. First, use model comparison and ensemble techniques to compare SARIMA and Prophet against advanced counterparts such as machine learning techniques as in [65], [66], [67]. Researchers can also explore more intricate time series models, such as state space models, VARs, and Bayesian structural models, for enhanced predictive accuracy. Anomaly detection within accident data can be explored, identifying unusual patterns and sudden spikes, which can help inform the development of early warning systems and targeted intervention strategies for more proactive accident prevention. The government of Ghana is also urged to support institutions like the MTTU and NRSC in terms of recruiting qualified personnel and providing logistics and quality education on road traffic accident prevention for the citizenry. The fight against RTA is the responsibility of every citizen. This research should be used to develop effective road safety strategies and policies, evaluate and monitor road safety initiatives' progress, and identify improvement areas. To enhance road safety and mitigate accidents, multifaceted approaches must be employed in road accident-related research in Ghana. These interventions span diverse domains, including infrastructure enhancement through improved road design and pedestrian/cyclist facilities; stringent enforcement of traffic regulations encompassing speed limits, seat belt and helmet laws, and measures against impaired driving; fostering public awareness through road safety campaigns and educational programs integrated into school curricula; elevation of vehicle safety standards through mandatory incorporation of advanced safety features and rigorous crash testing; establishment of comprehensive accident databases for data-driven decision-making and identification of accident patterns; legal and regulatory reforms about liability, insurance, and penalty structures, to bolster road safety. By integrating these measures, we aim to reduce the burden of road accidents on society and create a safer road environment in a low-middle income country such as Ghana.

## Funding statement

This research did not receive any specific grant from funding agencies in the public, commercial, or not-for-profit sectors.

## Additional information

No additional information is available for this paper.

## CRediT authorship contribution statement

**Edmund F. Agyemang:** Writing – review & editing, Writing – original draft, Validation, Software, Methodology, Investigation, Formal analysis, Data curation, Conceptualization. **Joseph A. Mensah:** Writing – original draft, Supervision, Project administration, Methodology, Investigation, Formal analysis. **Eric Ocran:** Writing – original draft, Visualization, Software, Methodology, Formal analysis. **Enock Opoku:** Writing – original draft, Software, Project administration, Investigation, Formal analysis. **Ezekiel N.N. Nortey:** Writing – review & editing, Methodology, Investigation, Formal analysis, Conceptualization.

## Declaration of Competing Interest

The authors declare that they have no known competing financial interests or personal relationships that could have appeared to influence the work reported in this paper.

## Data Availability

The data used to support the findings of this study are available from the corresponding author upon request and can also be assessed from the R codes available on GitHub repository at github.com/Agyemang1z/Road-Accidents.
